The article "Diagnostic value of Flash dual-source CT coronary artery imaging combined with dual-energy myocardial perfusion imaging for coronary heart disease" was published in 2014. Journal: Exp Ther Med.

# Diagnostic value of Flash dual-source CT coronary artery imaging combined with dual-energy myocardial perfusion imaging for coronary heart disease

**DOI:** 10.3892/etm.2014.1541

**Published:** 2014-02-13

**Authors:** RUI-PING ZHAO, ZHI-RU HAO, ZHI-JUN SONG

**Affiliations:** 1 Department of Cardiology, Central Hospital of Baotou, Baotou, Inner Mongolia 014040, P.R. China; 2 Department of Surgical Oncology, Central Hospital of Baotou, Baotou, Inner Mongolia 014040, P.R. China

**Keywords:** dual-source CT, coronary artery imaging, myocardial perfusion, coronary heart disease

## Abstract

The present study aimed to investigate the diagnostic value of Flash dual-source CT coronary angiography (DS-CTA) combined with dual-energy myocardial perfusion imaging (DS-CTP) for coronary heart disease (CHD), as a single-stage examination. A total of 60 patients with CHD underwent DS-CT examination, as well as coronary angiography (CAG), as the reference standard. The patients were divided into <50% and ≥50% stenosis groups based on their coronary angiograms. The sensitivity, specificity, positive predictive value, negative predictive value and accuracy of the method for diagnosing stenosis of ≥50% were evaluated via DS-CTA combined with DS-CTP. Of the 60 patients, 59 showed satisfactory results that conformed to the diagnostic requirements. Using CAG as the reference standard, the sensitivity, specificity and positive and negative predictive values of the Flash DS-CT results in the ≥50% vascular stenosis group were 83.7, 92.7, 88.9 and 89.1%, respectively. The respective values for DS-CTA combined with DS-CTP for diagnosing CHD were 94.2, 91.1, 88.0 and 95.8%. Therefore, the results obtained indicate that DS-CTA combined with DS-CTP has a high diagnostic value for CHD. DS-CT is advantageous for diagnosing and prognosticating CHD.

## Introduction

Coronary heart disease (CHD) is a common cardiovascular disease. The recent increasing incidence of the disease, as well as being a serious risk to human health, has led to CHD becoming a leading cause of mortality worldwide. CHD is myocardial damage caused by changes in coronary circulation, resulting in an imbalance between myocardial demand and coronary blood flow. CHD is caused by functional changes and organic diseases. Clinical exercise with ECG testing, ultrasound echocardiography and radionuclide myocardial scans are used to diagnose CHD. Coronary angiography (CAG) is considered the ‘gold standard’ for diagnosing CHD. However, it was previously found that the fine coronary angiographic observations of certain patients did not explain their recurrent angina, which may have resulted from tiny vascular lesions caused by defects in myocardial perfusion. Coronary macrovascular and microvascular disease lead to angina due to poor myocardial perfusion. Thus, myocardial perfusion has attracted significant attention (1). In 1929, Werner Forssmann self-administered the first cardiac catheterization procedure; the procedure has since developed rapidly and become one of the most important medical advances in the 20th century. Judkins improved several aspects of the catheterization, allowing its wide use in clinical CAG. The process involves puncture of a major blood vessel (e.g., the femoral or radial artery) using a percutaneous needle and then insertion of a small catheter into the heart. CAG accurately and intuitively shows all coronary arteries. However, inadequacies in the process remain. Firstly, the procedure is traumatic, invasive and entails a certain degree of risk, which prevents patients with no marked symptoms from readily undergoing such an examination. Secondly, understanding the structure of the vascular wall and the features of atheroma is challenging. Thirdly, the procedure may not provide pathological and physiological information, including myocardial perfusion, metabolism and tissue activity. Furthermore, it does not provide information about microangiopathy myocardial perfusion blood flow, as well as a simple operation. Therefore, a safe, effective and noninvasive screening method for diagnosing CHD and assessing myocardial perfusion requires development (2).

Advanced Flash dual-source CT (DS-CT) uses two sets of ball-tube detector systems. A post-processing workstation and the corresponding software are used to obtain images of myocardial perfusion and determine myocardial ischemia, while simultaneously obtaining a surface reconstruction diagram to evaluate the coronary arteries. Studies have shown that coronary imaging using Flash DS-CT has a success rate of 100%. Myocardial perfusion imaging also meets the demands of clinical diagnosis. Ruzsics *et al* (3,4) evaluated the coronary arteries and myocardial perfusion of 35 patients using dual-energy CT. Myocardial perfusion imaging using CAG and single photon emission computed tomography (SPECT) under dual-energy mode revealed a sensitivity of 84%, specificity of 84% and accuracy of 92% for diagnosing stenosis of >50%. The corresponding values for DS-CT and SPECT were 92, 92 and 93%, which indicated the potential of Flash DS-CT scans for comprehensively evaluating coronary vascular stenosis and myocardial perfusion. With the clinical application of a new generation of dual-energy CT, Flash DS-CT may complete coronary imaging and myocardial perfusion imaging at the same time, resulting in a limited amount of radiation exposure (4,5). As a noninvasive examination, Flash DS-CT has been widely used for screening and diagnosing suspected coronary artery diseases (6–8). DS-CT reveals the anatomy of coronary arteries, as well as exhibiting the regional myocardial perfusion of coronary lesions (9,10). The present study aimed to determine the accuracy of DS-CT coronary imaging and myocardial perfusion for diagnosing CHD.

## Materials and methods

### Inclusion criteria

This study was conducted in accordance with the Declaration of Helsinki and with approval from the Ethics Committee of the Central Hospital of Baotou (Baotou, China). Written informed consent was obtained from all participants. There were 60 subjects, consisting of 38 males and 22 females aged 36–75 years (54.25±7.02 years). All subjects had clinical considerations or known CHD and were patients of the Central Hospital of Baotou between 2010 and 2011. All patients underwent DS-CT examinations and had a body mass index of 23.2±4.5 kg/m^2^ and a heart rate between 55 and 78 bpm (64±8 bpm).

### Exclusion criteria

Patients with hypersensitivity to iodinated contrast material, serious arrhythmia, respiratory distress, serious liver and kidney dysfunctions and decompensated ventricular dysfunction were excluded from the study.

### Flash DS-CT

The time resolution of the Flash Spiral scanning technology (Flash DS-CT; Somatom Definition Flash, Siemens Healthcare, Erlangen, Germany) was 75 msec and the entire heart scan lasted 0.25 sec. The technology clearly depicts diameters ≥1.5 mm of two to three branches of the coronary artery, without controlling the patient’s heart rate, to accurately determine the degree of stenosis. Reconstruction of the images was divided into two parts, one for dual-source CT coronary angiography (DS-CTA) analysis and another for dual-source CT myocardial perfusion imaging (DS-CTP) analysis. The DS-CTA images were analyzed and vessel branches were regarded as single units, with two heart imaging physicians estimating the coronary arteries. The DS-CTP images were analyzed using the 17 segment method recommended by the American Heart Association (AHA) (11). Two specialized cardiac imaging physicians completed the DS-CTP evaluation. Myocardial perfusion was evaluated in terms of normal perfusion and perfusion defects. The combination of DS-CTA and DS-CTP was compared with CAG for diagnosing CHD, using the method by Kachenoura *et al* (12), to elucidate the correlation of coronary stenosis with the myocardial ischemic region. Coronary artery stenosis was diagnosed as ≥2 defects in myocardial segment perfusion in the DS-CTP image.

### CAG

CAG was conducted by experienced interventional physicians following the Judkins method (13), whereas the images were analyzed by two experienced cardiologists. Based on the AHA classification system, the right coronary artery (RCA) was divided into segments 1–4 (proximal, middle, distal and posterior descending artery, respectively). The left main branch (LM) was segment 5, whereas the left anterior descending artery (LAD) was divided into segments 6–10 (the proximal, middle, distal and the first and second diagonal branch, respectively). The left circumflex artery (LCX) was divided into segments 11 to 15 (circumflex artery nearly segments, middle, distal and first and second obtuse marginal branch, respectively). Stenosis was defined as ≥50% occlusion.

### Grouping and comparison

CAG was used to classify the patients into groups according to the degree of stenosis: <50% and ≥50%. It was also used as the reference standard for detecting stenosis of ≥50% and determined whether its positive coincidence rate corresponded with that of DS-CT coronary imaging. The sensitivity, specificity and accuracy of DS-CT for diagnosing CHD was calculated, as well as the diagnostic sensitivity, specificity, positive and negative predictive value of DS-CTA combined with DS-CTP for diagnosing CHD.

### Statistical analysis

Data were analyzed using SPSS version 17.0 (SPSS, Inc., Chicago, IL, USA). The measurement data are expressed as mean ± SD and the count data were analyzed using a χ^2^ test. P≤0.05 was considered to indicate a statistically significant difference. CAG was regarded as the reference standard. The sensitivity, specificity, positive predictive value and negative predictive value of Flash DS-CT for diagnosing vascular stenosis were calculated using the following formulae: Sensitivity = true positive results/(true positive results + false negative results); specificity = true negative results/(true negative results + false positive results); positive predictive value = true positive results/(true positive results + false positive results); and negative predictive value = true negative results/(true negative results + false negative results).

## Results

### General information

Of the 60 patients who underwent DS-CTA and DS-CTP, 1 case was excluded due to patient obesity which affected the image quality. The remaining 59 patients fulfilled the diagnostic requirements. The coronary angiograms of the 60 patients indicated that 86 of the 240 coronary arteries had ≥50% stenosis. Among the patients, 6 had one vascular lesion, 22 had two vascular lesions and 12 had three vascular lesions. The DS-CTA showed that 81 coronary arteries had stenosis of ≥50%, whereas DS-CTA combined with DS-CTP indicated 92 coronary arteries had stenosis of ≥50%.

### CAG and CT coronary imaging

The coronary angiograms of the 60 patients indicated that 86 of 240 vessels had stenosis of ≥50%. This degree of stenosis was observed in 12 vessels in the RCA, 34 in the LCX, 38 in the LAD and 2 in the LM. The results of DS-CTA indicated that 81 arteries had coronary stenosis of ≥50%, of which 14 vessels were in the RCA, 32 in the LCX, 34 in the LAD and 1 in the LM (Table I).

### DS-CT and catheter angiography

Using CAG as the reference standard, the results indicated that 86 coronary arteries had stenosis of ≥50%, whereas the results from DS-CTA indicated that 81 branches had stenosis of ≥50%. The diagnostic sensitivity, specificity and positive and negative predictive values of DS-CTA for stenosis of ≥ 50% were 83.7, 92.7, 88.9 and 89.1%, respectively. DS-CTA combined with DS-CTP diagnosed ≥50% stenosis in 92 coronary arteries and had diagnostic sensitivity, specificity and positive and negative predictive values of 94.2, 91.1, 88.0 and 95.8%, respectively (Table II; Fig. 1).

## Discussion

CAG is often considered the ‘gold standard’ for diagnosing coronary artery stenosis, however, its invasiveness limits its routine application. With the development of CT coronary imaging technology, particularly Flash DS-CT, CTA and CTP may be performed without increasing the radiation dose, as well as improving the accuracy of the diagnosis of coronary artery stenosis. The most accurate method for diagnosing CHD is to obtain coronary anatomical information and evaluate the changes in coronary artery hemodynamics (14). The results obtained in the present study for the diagnostic sensitivity, specificity and positive and negative predictive values of DS-CT for vascular stenosis of ≥50% were 83.7, 92.7, 88.9 and 89.1%, respectively. However, for DS-CTA combined with DS-CTP for CHD, the subsequent values were 94.2, 91.1, 88.0 and 95.8%, respectively. Therefore, it was shown that DS-CT had a high negative predictive value and specificity for diagnosing coronary artery stenosis, which is consistent with the findings of a previous international study (15). The high specificity indicates that DS-CT has a similar diagnostic reliability to CAG. It was also found that combining DS-CTA with DS-CTP further improved the diagnostic sensitivity and accuracy. However, the combination had a lower specificity than DS-CTA alone. Using DS-CTP, the coronary perfusion defect did not indicate luminal stenosis for supplying blood.

Three cases with normal coronary angiograms showed perfusion defects under DS-CTP. The recurrent angina of certain patients with normal coronary angiograms indicated that microvascular disease was caused by poor myocardial perfusion; thus, these patients were diagnosed with cardiac X syndrome (13,16). The etiology and symptoms also applied to numerous patients with normal CAG. The coronary angiograms of specific patients showed vascular stenosis, mild coronary lesions and critical lesions (stenosis of 50–70%). However, the myocardial perfusion imaging results of these patients were normal, which indicated that the stenoses did not diminish myocardial perfusion (16). Subsequent treadmill tests revealed positive results. One study showed that only a certain amount of exercise induced changes in coronary artery blood flow, which in turn caused abnormalities in myocardial perfusion; the myocardial perfusion defects were visible in the images (13). Blankstein *et al* (17) hypothesized that poor myocardial perfusion was due to significant stenosis of the coronary blood supply. Otherwise, the defect was a false positive (18). These studies (19) showed the mutual correlation and the inherent differences between morphological and functional examinations, which implied a correlation between stenosis and ischemia. The seriousness of local narrowing was insufficient to predict its effect on the dynamics of myocardial blood flow. Specific cases revealed inconsistencies between coronary anatomical narrowing and myocardial perfusion. Myocardial perfusion was directly associated with the symptoms, signs and prognosis of the patients. DS-CT was capable of diagnosing coronary artery stenosis, as well as revealing all types of myocardial perfusion defects. By combining morphological and functional information on the coronary circulation, the accuracy of CHD diagnosis may be increased, providing a reliable basis for the corresponding treatment. In conclusion, Flash DS-CTA combined with DS-CTP may reflect the two aspects of coronary atherosclerosis and myocardial ischemia, therefore allowing a more accurate identification of vessel lesions. The combination improved the accuracy of diagnosing CHD and stratifying the prognostic risks, which is likely to provide a reliable basis for further assessment of the clinical situation and prognosis to select the best treatment (20).

However, the present study had certain limitations. Firstly, the study involved a single institution only; accurately determining the diagnostic value of this imaging technology requires multicenter studies. Also, the sample size of the present study was relatively small and should be increased in future studies. Secondly, the DS-CTP scans were obtained with the patients in a resting state; further studies are required to be conducted in the drug-loading state.

Flash DS-CT is a single stage examination, overcoming the previous inability to simultaneously conduct CAG and myocardial perfusion imaging. However, the present study is prospective and in the initial stages. The current literature on this subject is limited; thus, the observations may not be clinically applied at present. Further studies are required to promote DS-CT cardiac imaging technology for comprehensively assessing patients with CHD or as a potential diagnostic method for high-risk patients.

## Figures and Tables

**Figure 1:** (A) Flash DS-CT, the nearly whole block of the proximal RCA. (B) CAG, the nearly whole block of the nearly RCA. (C) Flash DS-CT, defect of myocardial perfusion at the inferior wall. DS-CT, dual-source-CT; CAG, coronary angiography, RCA, right coronary artery.

**Table I:** Comparison of CAG and CT coronary imaging.

	≥50% stenosis (n)	
	
Lesion sites	CAG	CT
RCA	12	14
LCX	34	32
LAD	38	34
LM	2	1
Total	86	81

CAG, coronary angiography; RCA, right coronary artery; LCX, left circumflex artery; LAD, left anterior descending artery; LM, left main branch.

**Table II:** Coronary stenosis observed with DS-CT and catheter angiography.

		Catheter angiography	
		
CT technique	CT result	Positive	Negative
DS-CTA	Positive	72	9
	Negative	14	115
DS-CTA + DS-CTP	Positive	81	11
	Negative	5	113

DS-CTA, dual-source coronary angiography; DS-CTP, dual-source myocardial perfusion imaging.
